This article has been retracted.

# The impact of different plant extracts on population suppression of *Helicoverpa armigera* (Hub.) and tomato (*Lycopersicon esculentum* Mill) yield under field conditions

**DOI:** 10.1371/journal.pone.0260470

**Published:** 2021-12-01

**Authors:** Shahbaz Ali, Yunzhou Li, Inzamam Ul Haq, Waseem Abbas, Muhammad Zeeshan Shabbir, Muhammad Musa Khan, Mehmet Mamay, Yasir Niaz, Tahir Farooq, Milan Skalicky, Ali Tan Kee Zuan, Omaima Nasif, Mohamad Javed Ansari

**Affiliations:** 1 Department of Plant Pathology, College of Agriculture, Guizhou University, Guiyang, Guizhou, China; 2 Department of Agricultural Engineering, Khawaja Fareed University of Engineering and Information Technology, Rahim Yar Khan, Punjab, Pakistan; 3 Department of Plant Protection, College of Crop Protection, Gansu Agricultural University, Lanzhou, China; 4 Department of Entomology, University of Agriculture Faisalabad, Faisalabad, Pakistan; 5 Plant Protection Research Institute, Guangdong Academy of Agricultural Sciences, Guangzhou, Guangdong, China; 6 Key Laboratory Bio Pesticide Innovation and Application, Engineering Research Centre of Biological Control, South China Agriculture University, Guangzhou, P. R. China; 7 Department of Plant Protection, Faculty of Agriculture, Harran University, Şanlıurfa, Turkey; 8 Department of Botany and Plant Physiology, Faculty of Agrobiology, Food and Natural Resources, Czech University of Life Sciences, Prague, Czechia; 9 Department of Land Management, Faculty of Agriculture, Universiti Putra Malaysia, Selangor, Malaysia; 10 Department of Physiology, College of Medicine and King Khalid University Hospital, King Saud University, Medical City, Riyadh, Saudi Arabia; 11 Department of Botany, Hindu College Moradabad (Mahatma Jyotiba Phule Rohilkhand University Bareilly), India; Ghazi University, PAKISTAN

## Abstract

*Helicoverpa armigera* (Hub.) is a destructive pest of the tomato (*Lycopersicon esculentum* Mill) crop in Pakistan. Although insecticides are the primary management strategy used to control *H*. *armigera*, most of them are not effective due to considerable toxic residual effects on the fruits. Nonetheless, *H*. *armigera* is rapidly evolving resistance against the available pesticides for its management. This situation calls upon the need of alternative management options against the pest. Different plant extracts have been suggested as a viable, environment-friendly option for plant protection with minimal side effects. Furthermore, the plant extracts could also manage the insect species evolving resistance against pesticides. This study evaluated the efficacy of different plant extracts (i.e., Neem seed, turmeric, garlic and marsh pepper) against *H*. *armigera*. Furthermore, the impact of the plant extracts on growth and yield of tomato crop was also tested under field conditions. The results revealed that all plant extracts resulted in higher mortality of *H*. *armigera* compared to control. Similarly, the highest plant height was observed for the plants treated with the plant extracts compared to untreated plants. Moreover, the highest tomato yield was observed in plants treated with plant extracts, especially with neem seed (21.013 kg/plot) followed by pepper extract (19.25 kg/plot), and garlic extract 18.4 kg/plot) compared to the untreated plants (8.9 kg/plot). It is concluded that plant extracts can be used as eco-friendly approaches for improving tomato yield and resistance management of *H*. *armigera*.

## Introduction

Tomato (*Lycopersicon esculentum* Mill) is an important and the most popular vegetable crop, grown and eaten around the globe. Tomato ranks second among major vegetables grown in Pakistan [1]. It has become more popular and area under tomato cultivation is increasing gradually in the country [2]. Tomato was cultivate on was 60.7 thousand hectares with 566 thousand tones production in Pakistan during 2015 [3]. Pakistan is 37^th^ largest tomato producer in the world. However, country’s tomato production is low than developed countries in the world. Insect pests’ infestation is the major threat reducing tomato yield in Pakistan. Tomato crop is more likely to be attacked by several insect species from seedling to fruiting. *Helicoverpa armigera* (Hub.) is a destructive pest of tomato crop in Pakistan causing significant yield losses that worth 5 billion US$ annually [4]. The pest starts damaging leaves in the early growth stages and flowers are affected at later stage where the pest bores into the fruits, reducing their market value and making the fruits unfit for human consumption [5].

For decades, synthetic pesticides have been regarded as one of the most effective tools for pest management. Although pesticides are very effective and give quick results, their widespread use causes environmental pollution, human health risks, pollinator toxicity, pest revival, insect-pest resistance, secondary pest outbreaks, and residues in the food [6, 7]. Besides, intensive use of chemical pesticides have resulted in the evolution of insecticide resistance in *H*. *armigera* against commonly used insecticides [8]. This situation has necessitated the development of alternative insecticides which should be relatively inexpensive, effective in killing pests, and environment-friendly [9]. A promising alternative is to explore the plants with insecticidal properties for the development of botanical insecticides. Botanical insecticides have a great possibility to develop because Pakistan has a high diversity of plants that might contain active insecticide compounds.

Botanical insecticides are chemicals with insecticidal properties extracted from plants. Botanical insecticides allegedly cause little threat to the environment and almost none to plants, affect only targets insects, delay evolution of insecticide resistance, compatible with other pest control strategies, and produce healthy agricultural products free from synthetic insecticide [10]. The application of plant-based insecticides is useful in controlling caterpillars and is compatible with biological control techniques and biopesticides [11]. Several earlier studies have reported that plant extracts have successfully managed noxious insect pests [12–14].

The management of tomato insect pests has not been documented widely except using chemical pesticides. However, use of botanical extracts is a new approach for the management of tomato pests which has attained special attention of researchers worldwide. Many researchers have reported that botanical extracts have insecticidal [12–14] properties; thus, can be used for the control of agricultural pests. This can help to avoid environmental risks, environmental pollution, non-target effects caused by chemicals and beneficial for existing socioeconomic conditions. Although botanical pesticides have been studied in several laboratory tests [15], there are few studies that give findings from practical use, and biological efficacy against tomato fruit borer is lacking. In the light of above-mentioned background, the current study was conducted to infer the effect of different botanical extracts on *H*. *armigera* and yield contributing factors of tomato.

It was hypothesized that different plant extracts will differ in their efficacy of suppressing *H*. *armigera* infestation. Nonetheless, the application of all extracts would result in higher mortality compared to no application of extracts. It was further hypothesized that application of plant extracts will improve growth and yield attributes of tomato crop. The results would help to suppress the pest and improve tomato productivity with environment-friendly pest management option.

## Materials and methods

### Plant materials and growth conditions

Tomato plants were sown in sandy loam soil (pH: 6.7) at Entomological Research Area, Department of Entomology, University of Agriculture Faisalabad, Pakistan (31°26′2 N, 73°3′53.6′ E), during August 2018 and 2019. The mean temperature ranged from 28.6 to 34.5 °C and mean relative humidity ranged between 43.9 and 64.3% during the study period. The plant-to-plant and row-to-row distances were kept 30 and 65 cm, respectively. There were five rows and each row consisted of ten plants in each experimental unit. The size of each experimental unit was 26 m^2^. Standard agronomic practices recommended by the Agriculture Extension Department Government of Punjab, Pakistan for tomato crop were opted during both growing seasons.

### Experimental design and treatments

The experiment was arranged according to completely randomized design (CRD) with three replications. Four botanical extracts (i.e., Neem Seed, Turmeric, Garlic and Marsh Pepper) were applied and their efficacy was checked 3 and 7 days after application. In total, there were five treatments (4 botanical applications and one untreated control).

### Preparation of plant extracts

Neem seed, turmeric, garlic and marsh pepper were bought from local market (31°26′2 N, 73°3′53.6′ E), washed and dried under shade for 7 days. The dried plant parts were separately grinded into fine powder. For each plant a 10% stock solution was prepared by mixing 100 grams of powder in 1 liter of distilled water in a flask. The mixture was shaken properly, placed at room temperature for 24 hours and then filtered using a plain cloth to remove impurities.

### Application of plant extracts

For the application of plant extracts, tomato plants were sprayed twice at fifteen days interval using Knapsack sprayer after first fruiting. At the time of spray, polythene sheet was hanged around each plot to protect the adjacent plots from the drift effect. The infestation of *H*. *armigera* was recorded after 3 and 7 days of plant extracts application.

### Data collection

Mature tomato fruits were harvested from each experimental unit. Number of damaged fruits and weight of all harvested tomato fruits was recorded for each experimental unit. Total yield of each experimental unit was calculated by adding yield of tomato fruits per harvesting. Plant height in all the experimental units was measured using meter rod. The population reduction percentage was calculated by counting the number of insects in treated and untreated plots before and after the application of plant extracts.

### Statistical analysis

The collected data on measured traits were analyzed to infer the differences among growing seasons through paired t test, which indicated that year effect was non-significant. Therefore, data of both growing seasons were pooled for further analysis. The data were tested for normality using Shapiro-Wilk normality test, which indicated that data had a normal distribution. Hence, original data were used for further analysis. One-way analysis of variance (ANOVA) was used to test the significance in the data. The means were compared by least significant difference post hoc test at 5% probability where ANOVA indicated significant differences. The dataset of the manuscript has been given as S1 Dataset.

## Results

Different plant extracts significantly (F_2,14_ = 114.08, *P*<0.01) altered plant height of tomato plants (Table 1). The highest plant height (88.17±2.19 cm) was recorded for neem seed extract which was followed by marsh pepper extract (84.15±0.84 cm) and garlic extract (82.12±1.55 cm). The lowest plant height (66.48±0.91 cm) was recorded for control treatment of the study (Fig 1).

**Fig 1:** The impact of different plant extracts on plant height (cm) and yield (kg/plot) of tomato plants. The values are means ± SD (n = 3). Different lower-case letters on bars indicate significant differences among treatments at P<0.05.

**Table 1:** Analysis of variance for effect of natural insecticides on height (cm) and yield (Kg/plot) of tomato.

	Degrees of Freedom	Sum-of-Squares	Mean Square	F Value	P-Value
Plant height (cm)	4	887.270	221.817	114.08	0.0000*
Yield (kg/plot)	4	269.323	67.3307	159.64	0.0000*

* = significant

All the treatments significantly (F_2,14_ = 159.64, *P*<0.01) affected total yield of tomato plants. The highest yield (21.013±0.67 kg/plot) was noted for neem seed extract which was followed by marsh pepper extract and garlic extract, where yield per plot was 19.25±0.56 kg and 18.4±0.58 kg, respectively. The lowest yield (8.9±0.58kg) per plot was recorded in control treatment of the study (Fig 1).

Different plant extracts significantly (F_2,14_ = 140.76, *P*<0.01) affected the population of *H*. *armigera* three and seven days after treatment after both rounds of spray (Table 2). The highest reduction in Population (48.81 ± 4.28%) was recorded with neem seed extract followed by marsh pepper extract (43.177 ± 1.73%) and garlic extract (37.46 ± 2.78%). The lowest reduction in population was noted for control treatment where it was only 2.22 ± 1.92% (Fig 2).

**Fig 2:** Population reduction percentage of *H*. *armigera* larvae in first round of spray at 3 and 7 days after treatment (DAT) on tomato plants treated with foliar application of various plant extracts. The values are means ± SD (n = 3). Different lower-case letters on bars indicate significant differences among treatments at P<0.05.

**Table 2:** Analysis of variance for effect of natural insecticides on population reduction percentage of *H*. *armigera* after three and seven days of first and second round of spray.

Population Reduction percentage	Degree of Freedom	Sum of Squares	Mean Square	F value	P value
**First Round of Spray**					
Three days after treatment	4	4072.81	1018.20	140.76	0.0000*
Seven days after treatment	4	5497.66	1374.41	267.65	0.0000*
**Second Round of Spray**					
Three days after treatment	4	3994.75	998.68	165.97	0.0000*
Seven days after treatment	4	6183.26	1545.82	374.46	0.0000*

* = significant

The highest population reduction percentage (62.93 ± 1.38%) was recorded for neem seed extract after seven days of spray. The population reduction percentage after seven days in marsh pepper extract, garlic extract and turmeric extract was 59.22 ± 1.51%, 53.08 ± 1.08% and 40.683 ± 2.19%, respectively. The lowest population reduction after 7 days of application in first round of spray was 10.00 ± 3.33%, recorded for control treatment (Fig 2).

All plant extracts significantly (F_2,14_ = 165.97, *P*<0.01) affected the population of *H*. *armigera* in second round of spray at three days after treatment. The highest population reduction percentage (49.383 ± 2.69%) was observed for neem seed extract followed by marsh pepper and garlic extract, where population reduction was 48.237 ± 1.78% and 44.7 ± 1.79%, respectively. The lowest population reduction (5.55 ± 1.92%) was recorded in control treatment of the study (Fig 3).

**Fig 3:** Population reduction percentage of *H*. *armigera* larve in second round of spray at 3 and 7 days after treatment (DAT) on tomato plants treated with foliar application of various plant extracts. The values are means ± SD (n = 3). Different lower-case letters on bars indicate significant differences among treatments at P<0.05.

All plant extracts significantly (F_2,14_ = 114.08, *P*<0.01) affected the population of *H*. *armigera* seven days after the treatment during second round of spray. The highest population reduction percentage (73.69 ± 2.07%) was recorded for neem seed extract, followed by marsh pepper extract, garlic extract and turmeric extract, where population reduction was 67.077 ± 2.73%, 57.897 ± 2.01% and 50 ± 2.00%, respectively. The lowest population reduction (15.557 ± 1.93%) was recorded for control treatment of the study (Fig 3).

## Discussion

Different plant extracts, as hypothesized, significantly differed in their ability to suppress the population of *Helicovepa armigera*. Similarly, the applied extracts also differed in their ability to improve the growth and yield of tomato. The highest population reduction and the highest improvement in yield was noted for neem seed extract compared to the rest of the extracts included in the study. The control treatment recorded the highest population of *H*. *armigera* and yield of tomato. These results warrant that neem seed extract has the potential to be used as botanical insecticide against *H*. *armigera*. The differences in plant height can be linked to different number of insects feeding on tomato plants after spraying plant extracts. The plants with lower infestation faced no stress due to herbivory; thus, had higher plants compared to the plants under higher herbivory stress due to higher population of *H*. *armigera*. Results of current study indicate that the lowest plant height of tomato was recorded for control treatment where no plant extracts were applied. These results are in agreement with a previous study which reported that the highest plant height was noted for the plants treated with seed extract [16]. It is also reported that use of botanical extracts can considerably increase plant height and yield of tomato plants. Significantly increased plant height (37%) and more fruit yield (63%) was recorded in plants treated with higher concentrations of plant extracts mixed with fungicide [17]. The differences in yield are due to the different level of insect population after the spray of plant extracts. The application of plant extracts considerably reduced insect population. Findings of this study are in line with the results explained by Nisbet [18] where the highest yield was found with neem extract application. Similarly the lowest yield of tomato has been recorded for untreated control plants in another study [19]. It is also reported that when larval population of *H*. *armigera* is low, it increases the yield of potato. The present results are also in agreement with another finding who reported that profitable fruit yield was noted with the application of plant extracts as compared to untreated plots [20].

Azadirachtin-based compounds have insecticidal properties, and act as feed deterrents, and repellents. These compounds also have physiological properties such as decreasing survival, disturbing molting and also reproduction of insects [21]. Anti-feeding effect of garlic and onion reduced the ability of the insects or cutworms to feed [22]. Results of this study are in line with previous studies who reported that number of infested fruits was decreased when tomato plants were treated with neem oil at 3.0 m/L of water [16]. It is also reported that neem seed extracts and chemical pesticides had similarly effective in suppressing the population of *H*. *armigera* and saving crop from major insect damage [8]. Under laboratory conditions, percentage mortality of *H*. *armigera* larvae was increased when treated with neem extract as well as with neem + annona + mahua extract [23]. The number of larvae per plant were decreased when okra plants were treated with NSKE 5% [24]. Another study revealed that >68% reduction in *H*. *armigera* larvae was recorded at 7 and 14 days after the applications of neem seed extract [25]. Similarly, neem seed extract mixed with citronella oil performed better by decreasing per plant population of *H*. *armigera* larvae as reported by Subiyakto [9]. According to Yankanchi and Patil [26], 1% leaf extract of *V*. *negundo* dramatically reduced larval population of *H*. *armigera* in cabbage by 40%. Sahare et al. [27] discovered that alkaloids, saponin, and flavonoids are present in the leaf of *V*. *negundo* which are responsible for insecticidal activities. Previous research has found that *A*. *calamus* rhizome, *V*. *negundo* leaves, and *A*. *vasica* extracts contain alkaloids, tannins, saponins, phenolics, and flavonoids and extracts of these plants are efficient against *H*. *armigera* [28–33]. Mallapur and Ladaji [34] reported 56% reduction in *H*. *armigera* population in the treatment of *V*. *negundo*, *A*. *indica*, and *Aloe vera* extract. Mathuru and Mehta [35] reported that botanical insecticides based on extracts from *A*. *calamus* rhizome, *V*. *negundo* leaf, and *A*. *vasica* rhizome were superior than *D*. *deltoidea* tuber extract. According to Kumar and Prasad [36], 5% of extracts of *A*. *indica*, *A*. *calamus*, *V*. *negundo*, and *A*. *vasica* produced substantial mortality in *H*. *armigera*. Raja et al. [37] discovered that the active chemicals -asarone, cis-asarone, trans-asarone, and acoramone present in the rhizome extract of *A*. *calamus* have biological activity. Rastogi and Mehrotra [38] discovered vitricin, flavonoid-penducularisin, negundoside, and adhavasinone as active ingredients in the leaves of *V*. *negundo* and *A*. *vasica*. Aside from insecticidal, feeding deterrent, and growth suppressing activities, BI based on *A*. *calamus* and *V*. *negundo* have discovered benefits that promote product persistence [39]. Generally, *A*. *calamus* is critical for antifeedant, repellence, or deterrence for pest species. For example, extracts from the seed of *A*. *calamus* showed an antifeedant effect on *Spodoptera litura* [40].

## Conclusion

Based on current study, it was concluded that the use of botanical extracts is an alternative to synthetic insecticide as they are cheap, easily available and relatively safe to the natural enemies and other non-target species. Therefore, it is recommended to use different plant based indigenous botanical insecticides for the sustainable management of *H*. *armigera* in tomato and other crops.

## Supporting information

S1 Dataset (XLSX)
